The article "Medical Information Mining-Based Visual Artificial Intelligence Emergency Nursing Management System" was published in 2021. Journal: J Healthc Eng.

# Medical Information Mining-Based Visual Artificial Intelligence Emergency Nursing Management System

**DOI:** 10.1155/2021/4253606

**Published:** 2021-11-25

**Authors:** Aihua Dong, Jian Guo, Yongzhi Cao

**Affiliations:** ^1^Department of Emergency, The First Affiliated Hospital of Soochow University, Suzhou, Jiangsu 215006, China; ^2^Transfusion Center, The First Affiliated Hospital of Soochow University, Suzhou, Jiangsu 215006, China

## Abstract

This study aims to design a set of the visual artificial intelligence system based on medical information mining for hospital emergency care management. A visual artificial intelligence emergency first aid nursing management system is designed by analyzing the needs of the emergency first aid nursing management system. The results show that system personnel allocation, comparative management, record management, query management analysis, basic setup analysis, nursing management basis, and nonfunctional requirements all need to be optimized for the emergency first aid management system. In this study, the comparative management module, log management module, and the query management module are designed, and the emergency first aid management system of different APP terminal functions in different modules is described in detail. The nursing document query business is tested, and the corresponding time of query of nursing assessment sheet, nurse shift record, nurse record, and physical sign observation sheet is 375.50 ms, 351.48 ms, 336.36 ms, and 245.57 ms, respectively. It shows that the visual artificial intelligence emergency nursing management system based on medical information mining can provide convenience for clinical work to a large extent and has potential application value in hospital emergency nursing work.

## 1. Introduction

Medical information (MI) is a combination of medicine and computer science that aimed to facilitate the acquisition, storage, retrieval, and utilization of health and biomedical information [1]. As an emerging edge-cross discipline, it not only concerns computer and information technology but also uses clinical guidelines, corresponding medical terminology, and information exchange system as a platform [2]. In recent years, medical information mining technology has been increasingly valued in medical-related departments and extensively used in many fields [3]. Medical information includes clinical electronic medical records, basic hospital information systems, clinical disease decision support systems, image information extraction technology, and telemedicine [4]. With the widespread application of electronic medical records and the digitization of medical equipment and instruments, the information capacity of hospital databases has continued to expand [5]. Data standards include two types, namely, information standards and text standards. The text standard means that the standard must be expressed in the form of text and not in the form of pictures. It is generally called a medical data system and includes a series of words with specific meanings [6]. It contains the human and veterinary medical system terminology standard SNOMED formulated by the American Pathology Association and the medical system terminology standard read codes developed by the British Health Center [7]. Nowadays, the most commonly used information standard is called Health Level 7 (HL7), also known as a standard health information transmission protocol, including DICOM [8], and it facilitates the exchange of hospitalization data between the laboratory system and the electronic medical record system.

The article "Medical Information Mining-Based Visual Artificial Intelligence Emergency Nursing Management System" was published in 2021. Journal: J Healthc Eng.

The medical treatment of the emergency department is the key of the key in the hospital. The emergency department mainly serves to patients with acute and severe diseases, and the diagnosis and treatment level of this department is directly related to the quality of life of patients in the later period and the degree of satisfaction of patients with the hospital. However, the large flow of emergency patients and the high management cost and the difficulty of emergency care require the rational allocation of resources of the emergency department. Buscema M used automatic compressed mapping (Auto-CM) to find out the subtle associations between various variables [9]. This method can guarantee the adaptive strength of the connection between any dataset and all related variables. Based on the limited medical information data, the artificial intelligence neural network can effectively predict the bone metastasis of prostate cancer patients [10]. Scholars have used the artificial intelligence-based first aid priority management system to improve the quality and satisfaction of the care for patients in the emergency department [11].

Then, a visual artificial intelligence nursing system is developed. It has functions of comparative management, query management, record management, nursing document management, basic settings, and basic nursing management, which are mainly realized through an APP end [12, 13]. The system uses the design model of Model View Controller (MVC), the MyBatis framework, and other technologies [14]. Studies have shown that the MVC model has many standardized hierarchical frameworks concerning technologies such as the MyBatis framework and Oracle database [14]. The MyBatis framework includes multiple interfaces, such as data management and mapper [15].

The article "Medical Information Mining-Based Visual Artificial Intelligence Emergency Nursing Management System" was published in 2021. Journal: J Healthc Eng.

Above all, this study focuses on the design of the medical information visualization emergency first aid system. With first aid measures in hospital emergency departments as the breakthrough point, the work procedures of the nurse, head nurse, and nurse directors are analyzed. According to specific requirements, the APP end of the emergency first aid management system is designed, and the submodules of the visual artificial intelligence emergency first aid management system are described in detail. Finally, the system is tested. The study provides a more practical management system for hospital emergency nursing and convenience for clinical work and improves the work efficiency of medical workers.

## 2. Establishment of the Apriori Optimization Algorithm

### 2.1. Probabilistic Interest Model

The probability-based interest model algorithm is as follows:

(1) $$\begin{array}{c} \text{Int}\left(X⟶Y\right)=\frac{1-P\left(Y\right)}{\left(1-P\left(X\right)\right)\left(1-P\left(Y/X\right)\right)}, \end{array}$$

where *P*(*X*) represents the probability that transaction *X* appears in transaction set *D*.

(2) $$\begin{array}{c} P\left(X\right)=\frac{\text{Count}\left(X\right)}{N}. \end{array}$$

*P*(*Y*) represents the probability that transaction *Y* appears in food set *D*.

(3) $$\begin{array}{c} P\left(Y\right)=\frac{\text{Count}\left(Y\right)}{N}. \end{array}$$

*P*(*Y*/*X*) represents the probability of simultaneous occurrence of transactions *X* and *Y* in transaction set *D*.

(4) $$\begin{array}{c} P\left(\frac{Y}{X}\right)=\frac{\text{Count}\left(X\cup Y\right)}{N}. \end{array}$$

### 2.2. Differential Interest Model

The interest model based on differences is as follows.

(5) $$\begin{array}{c} \text{Int}\left(X⟶Y\right)=\frac{\text{Conf}\left(X⟶Y\right)-\text{Supp}\left(Y\right)}{\text{MAX}\left(\text{Conf}\left(X⟶Y\right)\right),\text{Supp}\left(Y\right)}, \end{array}$$

where MAX(Conf(*X*⟶*Y*)), Supp(*Y*) is an evaluation standard, which is used to ensure that Int(*X*⟶*Y*)<1 is established.

### 2.3. Related Interest Model

The interest model based on correlation is as follows.

(6) $$\begin{array}{c} \text{Int}\left(X⟶Y\right)=\frac{\text{Supp}\left(X\cup Y\right)}{\text{Supp}\left(X\right)\text{Supp}\left(Y\right)},\\ \text{Supp}\left(X\cup Y\right)=\frac{\text{Count}\left(X\cup Y\right)}{N},\\ \text{Supp}\left(X\right)=\frac{\text{Count}\left(X\right)}{N},\\ \text{Supp}\left(Y\right)=\frac{\text{Count}\left(Y\right)}{N}. \end{array}$$

The degree of interest based on relevance Int(*X*⟶*Y*) illustrates the relationship between the preceding and subsequent items *X* and Y in the association rule (*X*⟶*Y*).

### 2.4. Information Volume Interest Degree Model

The information-based interest model is as follows.

(7) $$\begin{array}{c} \text{Int}\left(X⟶Y\right)=P\left(X\right)\left[P\left(\frac{Y}{X}\right)\log\left(\frac{P\left(Y/X\right)}{P\left(Y\right)}\right)+1-P\left(\frac{Y}{X}\right)\log\left(\frac{1-P\left(Y\right)}{1-P\left(Y\right)}\right)\right],\\ P\left(X\right)=\frac{\text{Count}\left(X\right)}{N},\\ P\left(Y\right)=\frac{\text{Count}\left(Y\right)}{N},\\ P\left(\frac{Y}{X}\right)=\frac{\text{Count}\left(X\cup Y\right)}{N}. \end{array}$$

The interest degree model based on the amount of information comprehensively considers the conciseness of the association rule (*X*⟶*Y*), the amount of information, and the similarity of the probability distributions of the preceding item *X* and the subsequent item *Y*, and the probability of the preceding item is used as a measure of the conciseness of the preceding item of the association rule.

The article "Medical Information Mining-Based Visual Artificial Intelligence Emergency Nursing Management System" was published in 2021. Journal: J Healthc Eng.

### 2.5. Interest Model Based on Influence

The influence-based interest model is as follows.

(8) $$\begin{array}{c} \text{Int}\left(X⟶Y\right)=\log\frac{\text{Conf}\left(X⟶Y\right)/\text{Conf}\left(X⟶Y1\right)}{\text{Supp}\left(Y\right)/\text{Supp}\left(Y1\right)},\\ \text{Conf}\left(X⟶Y1\right)=\frac{\left(N-\text{count}\left(X\cup Y\right)\right)}{\text{Count}\left(X\right)},\\ \text{Supp}\left(Y\right)=\frac{\text{Count}\left(Y\right)}{N},\\ \text{Supp}\left(Y1\right)=\frac{\left(N-\text{count}\left(Y\right)\right)}{N}. \end{array}$$

### 2.6. Improved Algorithm

Through the comparison and analysis of various interest degree models, as well as the mining of medical information, the improved algorithm is as follows.

(9) $$\begin{array}{c} \text{Int}\left(X⟶Y\right)=\text{Conf}\left(X⟶Y\right)-\text{Conf}\left(X1-Y\right),\\ \text{Int}\left(X⟶Y\right)=\frac{P\left(X\cup Y\right)}{P\left(X\right)}-\frac{P\left(X1\cup Y\right)}{P\left(X1\right)},\\ \text{Int}\left(X⟶Y\right)=\frac{P\left(X\cup Y\right)-P\left(X\right)P\left(Y\right)}{P\left(X\right)\left[1-P\left(X\right)\right]}. \end{array}$$

## 3. Requirement Analysis of the Visual Artificial Intelligence Emergency Nursing Management System

### 3.1. System Requirements Analysis

There are many problems in the hospital emergency nursing system. Nurses are not efficient in the processes of infusion and dispensing, and it is difficult for nurses to quickly query the patient's basic information, doctor's orders, and other medical information in their daily work. There lacks an effective way to manage nursing document information, and basic nursing management also has various shortcomings. Therefore, a visual nursing system for the emergency department based on artificial intelligence is developed in the form of an APP. The system requirements are shown in Figure 1.

The article "Medical Information Mining-Based Visual Artificial Intelligence Emergency Nursing Management System" was published in 2021. Journal: J Healthc Eng.

In the APP end of the medical information-based visual artificial intelligence emergency nursing system, many new services have been added to meet the various needs of nurses, such as management of prescribing, infusions, and doctor orders; in record management module, nurses can view and deal with physical signs and documents; the query management module includes patient information, medical order information, and treatment of patients; and statistical performance, monitoring of nursing links, and application settings are included in the basic settings module. The business flowchart of the visual artificial intelligence emergency nursing management system based on medical information is shown in Figure 2.

### 3.2. System Personnel Allocation

The visual artificial intelligence emergency nursing management system includes nurses, head nurses, and nursing department. The system APP enables the operator to carry out a series of operations, such as comparison, query, and record management. The roles involved in the of emergency nursing management system are shown in Figure 3.

### 3.3. Requirements Analysis on the APP of the Visual Artificial Intelligence Emergency Nursing Management System Based on Medical Information Mining

#### 3.3.1. Comparison Management

In the functional section of the APP, nurses in the emergency department can enter the comparison management interface through the APP to process fluid dispensing and infusion-related services to achieve rapid emergency nursing. The comparison management module is shown in Figure 4.

#### 3.3.2. Record Management

The record management module reflects a series of nursing-related requirements, and it can collect nursing signs, record nursing sign information, generate nursing documents, process document information, and manage nursing measures. The record management module is shown in Figure 5.

#### 3.3.3. Query Management Analysis

The query business concerns patient information, doctor's order information, and diagnosis and treatment expenses. The basic information above can be obtained through query module. The query management module is shown in Figure 6.

#### 3.3.4. Basic Setting Analysis

The basic setting module reflects the relevant needs of statistical nursing work, monitors nursing links, and obtains notifications. In addition, users can also set according to their own habits, such as signature keyboard, automatic data reference, and writing input. The basic setting analysis module is shown in Figure 7.

#### 3.3.5. Basic Nursing Management

Basic nursing management involves basic management businesses, including nursing document management, human resource management, nursing quality management, adverse event management, and nursing statistical analysis. The basic nursing management module is shown in Figure 8.

The article "Medical Information Mining-Based Visual Artificial Intelligence Emergency Nursing Management System" was published in 2021. Journal: J Healthc Eng.

### 3.4. Nonfunctional Requirements

The visual artificial intelligence emergency nursing management system based on medical information mining puts forward higher requirements for adaptability and safety. Adaptability: the mobile service components of the system should have large memory storage and can adapt to the complex and changeable use environment. Safety: due to irresistible factors such as slow network communication speed, mobile users will encounter poor communication or slow speed when logging in; in order to ensure the security of user logging in, the system should identify users who are offline multiple times in per unit time. Ease of use: the hospital has a large number of object-oriented nursing tasks of complex types. Therefore, the system should be able to provide a personalized setting system, so that nurses can flexibly set up according to their own operating habits.

## 4. The APP End of the Visual Artificial Intelligence Emergency Nursing Management System Based on Medical Information Mining

### 4.1. Design of the Comparison Management Module

Comparison management window and comparison management business are the basic categories of comparison management modules. The business category includes liquid dispensing management business, infusion management business, specimen collection business, medical order execution business, and liquid preparation entity, infusion management entity, specimen collection entity, and medical order execution entity. The comparison management design is given in Table 1.

The nurse sends an application for processing the preparation business. The system accepts the processing application, sequentially calls the comparison management window and business categories, and returns to the liquid preparation business. The processing of the liquid to be dispensed is shown in Figure 9.

### 4.2. Record Management Design

The functional category of the record management module includes record management window, record management business, nursing physical sign management business, nursing document management business, patrol management business, and nursing measure management business. The record management design is given in Table 2.

### 4.3. Query Management Design

The query management module includes query management window, query management business, patient information management business, medical order management business, diagnosis and treatment expense management business, and special patient management business. The entity category includes patient information entity type, diagnosis and treatment expense entity type, inspection and examination entity type, special patient entity type, and doctor order entity type. The query management design is given in Table 3.

The article "Medical Information Mining-Based Visual Artificial Intelligence Emergency Nursing Management System" was published in 2021. Journal: J Healthc Eng.

### 4.4. Basic Setting Design

The basic setting module includes basic setting window, basic setting business, performance statistics business, nursing link monitoring business, information push business, application setting business, nursing link entity, information entity, and performance statistics entity. The design of basic setting is given in Table 4.

The monitoring business in the nursing link is shown in Figure 10.

## 5. System Test

System test environment: Windows Server 2012 operating system, 1 TB hard disk, 4G processing memory; the Web server runs Windows 7 and has 500 GG hard disks and 2G processing memory; the browser kernel is IE and Safari; the APP terminal is the Android 5.0 operating system and can connect to the WiFi network. On the basis of formulating test cases, the test process is standardized, striving for the accuracy of system test results.  Figure 11 shows the test results of the comparative management module. The system does not execute the mixing task and the processing result information of the mixing.

Figure 12 shows the test results of nursing document query business. The corresponding time of query of nursing assessment sheet, nurse shift record, nurse record, and physical sign observation sheet is 375.50 ms, 351.48 ms, 336.36 ms, and 245.57 ms, respectively.

## 6. Discussion

In the study, the requirements on the visual artificial intelligence emergency nursing system are analyzed. Then, the role of the system is analyzed, each functional module is established, and the functional requirements are analyzed. As for the system design, the overall functional architecture of the system is designed.

The development of the APP adopts the MVC design pattern, Spring MVC framework, and other technologies. The MVC design pattern stipulates the responsibilities of the components and reduces the coupling between the components [16]. The use of the MyBatis framework brings complete data encapsulation and optimizes the data processing process [17]. The Spring MVC framework includes a perfect client request processing system, which is composed of components such as HandlerMapping and ViewReSolver. On the basis of integrating multiple modules, it enhances the display effect [18]. The APP of the visual nursing system realizes functions such as comparison management, record management, query management, and basic settings [19]. Comparison management window and comparison management business are the basic categories of comparison management modules. The business category includes liquid dispensing management business, infusion management business, specimen collection business, medical order execution business, and liquid preparation entity, infusion management entity, specimen collection entity, and medical order execution entity. The functional category of the record management module includes record management window, record management business, nursing physical sign management business, nursing document management business, patrol management business, and nursing measure management business. The query management module includes query management window, query management business, patient information management business, medical order management business, diagnosis and treatment expense management business, and special patient management business. The entity category includes patient information entity type, diagnosis and treatment expense entity type, inspection and examination entity type, special patient entity type, and doctor order entity type. The basic setting module includes basic setting window, basic setting business, performance statistics business, nursing link monitoring business, information push business, application setting business, nursing link entity, information entity, and performance statistics entity [20, 21]. The Apriori algorithm is an information mining algorithm for association rules, mainly used in the medical field. Its main idea is the two-stage frequency collection. It is mainly to search for *n* + 1 item through *n* items. This method is mainly divided into two steps, which are called connection steps and pruning steps [22, 23].

The article "Medical Information Mining-Based Visual Artificial Intelligence Emergency Nursing Management System" was published in 2021. Journal: J Healthc Eng.

## 7. Conclusion

In the study, the steps of emergency nursing and the needs in the process of emergency nursing are analyzed. It is found that there is a lack of effective means for nurses to compare the information of infusion and liquid dispensing. It is difficult for nurses in daily work to quickly query the patient basic information, such as orders, and the head nurse and nursing managers on lack of systematic methods of management for nursing documents information. Based on these problems, the visualization APP emergency care management system is designed and tested. The results show that the visual artificial intelligence first aid nursing management system APP designed in this study has certain operability, but there are still some limitations in this study. In this study, only APP window is designed, without Web window application. In subsequent studies, Web window design should be added to meet the needs of more functions. In conclusion, this study promotes the application of the artificial intelligence-based visual nursing system for hospital emergency care in clinical work, which provides convenience for clinical work and improves the work efficiency of medical workers.

The article "Medical Information Mining-Based Visual Artificial Intelligence Emergency Nursing Management System" was published in 2021. Journal: J Healthc Eng.

## Figures and Tables

**Figure 1:** Visual artificial intelligence emergency nursing management system.

**Figure 2:** The business flowchart of the visual artificial intelligence emergency nursing management system.

**Figure 3:** Personnel allocation of the visual artificial intelligence emergency nursing management system.

**Figure 4:** The comparison management module of the emergency nursing management system.

**Figure 5:** Record management module of the emergency nursing management system.

**Figure 6:** Query management module of the emergency nursing management system.

**Figure 7:** The basic setting analysis of the emergency nursing management system.

**Figure 8:** The basic nursing management module of the emergency nursing management system.

**Figure 9:** The processing sequence of the liquid to be dispensed.

**Figure 10:** Flowchart of the monitoring business in nursing link.

**Figure 11:** Comparison of management test results.

**Figure 12:** System performance test diagram.

**Table 1:** Comparison management design.

Type	Method
Liquid preparation	To-be-dispensed task query, to-be-dispensed task view, to-be-dispensed task processing, and to-be-dispensed task check
Infusion management	To-be-dispensed task query, to-be-dispensed task view, to-be-dispensed task processing, and to-be-dispensed task check
Specimen collection	Specimen collection, specimen viewing, specimen query, specimen query, and specimen modification
Medical order execution	Doctor's order query, doctor's order view, and doctor's order execution

**Table 2:** Record management design.

Type	Method
Nursing sign management	Nursing sign record, nursing sign submission, nursing sign modification, nursing sign review, and nursing sign printing
Nursing document management	Nursing document generation, nursing document viewing, nursing document printing, and nursing document query
Tour management	Tour record, tour query, tour view, tour processing, and tour print
Nursing measures management	Nursing measure formulation, nursing measure review, nursing measure query, nursing measure printing, and nursing measure modification

**Table 3:** Design of query management.

Type	Method
Patient information management	View patient information, query patient information, view admission records, view the first course of illness, and view course records
Medical order management	Doctor's order query, doctor's order view, and doctor's order processing
Management of medical expenses	Diagnosis and treatment cost statistics, diagnosis and treatment cost query, and diagnosis and treatment cost view
Inspection management	Inspection query, inspection review, and inspection processing
Special patient management	Hospital-wide patient review, fever patient review, pain patient review, special patient consultation, and special patient treatment

The article "Medical Information Mining-Based Visual Artificial Intelligence Emergency Nursing Management System" was published in 2021. Journal: J Healthc Eng.

**Table 4:** Design of basic setting.

Type	Method
Performance statistics	Nursing staff workload statistics, medical order execution statistics, patient inspection statistics, nursing operation statistics, nursing record statistics, and nursing document statistics
Nursing link monitoring	Check for unexecuted links, check for start links, check for pause links, and check for finished links
Information notification service	Information query, information view, and information push
Application settings business	Basic settings, data reference settings, batch entry settings, automatic reminder settings, and toolbox settings

## Data Availability

The data used to support the findings of this study are available from the corresponding author upon request.
